# A Novel Copper Chelate Modulates Tumor Associated Macrophages to Promote Anti-Tumor Response of T Cells

This article has been retracted.

**DOI:** 10.1371/journal.pone.0007048

**Published:** 2009-09-16

**Authors:** Shilpak Chatterjee, Ananda Mookerjee, Jayati Mookerjee Basu, Paramita Chakraborty, Avishek Ganguly, Arghya Adhikary, Debanjan Mukhopadhyay, Sudipta Ganguli, Rajdeep Banerjee, Mohammad Ashraf, Jaydip Biswas, Pradeep K. Das, Gourisankar Sa, Mitali Chatterjee, Tanya Das, Soumitra Kumar Choudhuri

**Affiliations:** 1 Department of In Vitro Carcinogenesis and Cellular Chemotherapy, Chittaranjan National Cancer Institute, Kolkata, India; 2 Department of Surgical Oncology, Hospital Unit, Chittaranjan National Cancer Institute, Kolkata, India; 3 INSERM, U-563, CHU Purpan, Toulouse, France; 4 Department of Molecular Medicine, Bose Institute, Kolkata, India; 5 Department of Pharmacology, Institute of Post Graduate Medical Education and Research, Kolkata, India; 6 Rajendra Memorial Research Institute of Medical Sciences, Patna, India; Harvard Institute of Medicine, United States of America

## Abstract

**Background:**

At the early stages of carcinogenesis, the induction of tumor specific T cell mediated immunity seems to block the tumor growth and give protective anti-tumor immune response. However, tumor associated macrophages (TAMs) might play an immunosuppressive role and subvert this anti tumor immunity leading to tumor progression and metastasis.

**Methodology/Principal Findings:**

The Cu (II) complex, (chelate), copper N-(2-hydroxy acetophenone) glycinate (CuNG), synthesized by us, has previously been shown to have a potential usefulness in immunotherapy of multiple drug resistant cancers. The current study demonstrates that CuNG treatment of TAMs modulates their status from immunosuppressive to proimmunogenic nature. Interestingly, these activated TAMs produced high levels of IL-12 along with low levels of IL-10 that not only allowed strong Th1 response marked by generation of high levels of IFN-γ but also reduced activation induced T cell death. Similarly, CuNG treatment of peripheral blood monocytes from chemotherapy and/or radiotherapy refractory cancer patients also modulated their cytokine status. Most intriguingly, CuNG treated TAMs could influence reprogramming of TGF-β producing CD4^+^CD25^+^ T cells toward IFN-γ producing T cells.

**Conclusion/Significance:**

Our results show the potential usefulness of CuNG in immunotherapy of drug-resistant cancers through reprogramming of TAMs that in turn reprogram the T cells and reeducate the T helper function to elicit proper anti-tumorogenic Th1 response leading to effective reduction in tumor growth.

## Introduction

Tumor cells escaping from the immune surveillance in immunocompetent individuals reflects inadequate function of the immune system. Induction of tumor specific T cell mediated immunity may block the tumor growth and may give protective anti-tumor immune response [1], [2]. However strong immune suppression in the tumor microenvironment makes the situation more complicated [3], [4]. It has been suggested that the growing tumors produce various chemoattractants that have been implicated in recruitment of monocytes in the tumor site. When monocytes are recruited into the growing tumor site, local cytokine milieu modulates the immunological functions of these newly recruited monocytes and educates them towards tumor-associated macrophages (TAMs) that are immunosuppressive in nature [5], [6], [7]. TAMs promote tumor cell proliferation and metastasis by secreting a wide range of growth and proangiogenic factors as well as various metalloproteinases [8], [9]. TAMs also possess poor antigen presenting ability and effectively suppress the induction of proper anti-tumor T cell response through the production of immunosuppressive cytokines like TGF-β and IL-10 [6], [10], as well as promote induction and infiltration of CD4^+^CD25^+^FoxP3^+^ T cells (Treg) at the tumor site [11]. However, evidence suggested that phenotype of TAMs can be reprogrammed and the presence of IL-12 in its local milieu plays key role in reprogramming of their functional cytokine profile towards proimmunogenic (IL-12 secreting) nature [12]. IL-12 also dictates the orchestration of T cell response towards generation of protective anti tumor response by stimulating T cells and NK cells to produce IFN- γ (13, 14, 15). Induction of IFN- γ production and suppression of IL-4 production by IL-12 has been shown to induce anti-tumor response in murine tumor models [14], [16]. Thus, if TAMs possess functional plasticity, it would be useful target for anti-tumor therapy because skewing them again towards proimmunogenic nature could induce proper anti tumor Th1 response that can effectively reduce tumor growth and metastasis.

It has been reported earlier that copper homeostasis plays a vital role in drug resistance in cancer and also found to be essential in mediating several intracellular signals in macrophage [17], [18]. An elevated copper level in macrophage is associated with the production of inflammatory cytokines whereas a copper deficiency attenuates its conventional immunological functions [19]. Previously our laboratory had synthesized a novel copper chelate [Copper N-2(hydroxy acetophenon) glycinate (CuNG)] which was found to be a potent immunomodulator able to elevate the number of CD4^+^ IFN-γ producing cells in drug resistant tumor [Doxorubicin resistant Ehrlich Ascites Carcinoma (EAC/Dox)] bearing mice [20], [21]. In this study we found that CuNG has direct effect on TAMs and can modulate their functional cytokine pattern, inducing their conversion from immunosuppressive to proimmunogenic nature. Herein we have also found that change in regulatory cytokine profile of TAMs was able to redirect the T helper function, reprogram Treg population and augment the induction of protective immune response in EAC/Dox bearing mice. Similar results were also obtained in case of peripheral blood monocytes from chemo and/or radiotherapy refractory patients.

## Results

### CuNG treatment can directly modulate the regulatory cytokine profile of Tumor Associated Macrophages (TAMs)

Previous study with the novel copper chelate CuNG revealed its immunomodulatory properties in EAC/Dox bearing mice. CuNG caused augmentation of apoptogenic inflammatory cytokine (mainly IFN-γ) production and resolution of tumors [21]. This finding prompted us to further investigate how this copper chelate (CuNG) induces the production of such inflammatory cytokines. First we have tried to know whether CuNG can directly act on CD4^+^ T cells [as this population is the predominant source of inflammatory cytokines following CuNG administration (i.m) [21]] to induce IFN-γ production. It was observed that in vitro application of CuNG did not have any significant effect in the IFN-γ production by CD4^+^ T cells obtained from EAC/Dox bearing mice (Fig. 1A). TAMs play pivotal role in suppression of IFN-γ producing CD4^+^ T cells (Th1 response) at the tumor site through establishment of immunosuppressive cytokine environment [22]. Therefore, we probed whether CuNG could modulate the functional behavior of TAMs from suppressive to proimmunogenic type so that protective Th1 response can be elicited. To test this possibility, EAC/Dox bearing mice were treated with CuNG (i.m, 5 mg/kg of body weight), TAMs were isolated 15 days following CuNG treatment (i.e., when tumors start to reduce prominently) and intracellular cytokine profile was checked by flow cytometry (Fig. 1B). It was observed that TAMs isolated from CuNG treated group released elevated level of IL-12 compared to the TAMs obtained from untreated EAC/Dox bearing mice (77.36% vs. 22.6%, MFI: 71.89±1.24 vs. 15.35±1.42). On the other hand, production of two major suppressive cytokines, IL-10 (63.21% vs. 94.09%, MFI: 48.68±0.95 vs. 82.44±0.68) and TGF-β (19.21% vs. 70.68%, MFI: 14.77±0.72 vs. 92.35±0.81) was found to be down regulated in the CuNG treated group compared to the untreated control.

**Figure 1:** Both in vitro and in vivo CuNG treatment caused alteration of cytokines profile of TAMs. A) ELISA. B) Flow cytometry. C) Fluorometric analysis. D, E & F) ELISA. In vitro CuNG treatment (2.5 µg/ml) did not change IFN-γ production from CD4^+^ T cells of TALs of untreated EAC/Dox bearing mice (A). TAMs were purified from peritoneal ascitic fluid of both untreated and 15 days of CuNG treated EAC/Dox bearing mice and labeled with anti F4/80 antibodies and with either intracellular IL-10 or IL-12 or TGF-β or with specific isotype control Abs. Immunofluorescence analysis were performed by flow cytometry. Representative data of 3 independent experiments is presented (B). Purified TAMs were either kept untreated or treated with CuNG in vitro and ROS was measured [in terms of peroxide using dichlorofluorescein diacetate (DCF-DA)] at different time points. Results are presented as mean±SD of 3 independent experiments (C). Purified TAMs from untreated EAC/Dox bearing mice were plated (2×10^6^ cells/500 µl). Cells were either kept untreated or pretreated with tocopherol (50 µM) for 1 h. Then the cells were further cultured for 12 h, 24 h and 48 h in the presence or absence of CuNG (2.5 µg/ml). The culture supernatants were collected and analyzed for cytokines IL-10 (D), IL-12 (E) and TGF-β (F) by ELISA and results are presented as mean±SE of 3 independent experiments, each experiment having every measurement in triplicate.

The result was further confirmed by performing ELISA for IL-12, IL-10 and TGF-β. It was observed that 12 h and 24 h cultures of TAMs in the presence of CuNG did not show any modulation in regulatory cytokine production but 48 h of CuNG treatment caused significant up regulation in IL-12 production (Fig. 1E) (>13.5 fold) whereas the suppressive cytokine TGF-β (Fig. 1F) production was highly (∼17.2 folds) and IL-10 production (Fig. 1D) was moderately down regulated (∼3.71 folds) as compared to the untreated control. These results together indicate that CuNG treatment significantly modulates the production of regulatory cytokines by TAMs.

Interestingly, it was observed that CuNG treated TAMs maintain a sustained higher level of reactive oxygen species (ROS; measured in terms of peroxide) till 18 h post treatment compared to untreated TAMs (Fig. 1C). Chelation of ROS with the anti-oxidant tocopherol (50 µM) reversed the nature of CuNG treated TAMs by increasing IL-10 and TGF-β production and decreasing IL-12 generation to levels comparable to untreated TAMs (Fig. 1D, E and F).

### In vivo administration of CuNG in EAC/Dox bearing mice induce Th1 type response

It has well been documented that the cytokine IL-12 plays a pivotal role in Th1 polarization [13], [15]. Since administration (i.m) of CuNG in EAC/Dox bearing mice induce elevated level of IL-12 production by TAMs at the tumor microenvironment, we therefore checked whether in vivo CuNG treatment could modulate the cytokine profile of the tumor associated lymphocytes (TAL) towards Th1 type. Flow cytometric analysis revealed that CD4^+^ population of TAL from CuNG treated group showed higher percentage of IFN-γ positive population compared to untreated group (21.42% vs. 3.54%). On the contrary, the percentage of IL-4 and TGF-β positive populations in TALs isolated from in vivo CuNG treated animals was found to be greatly reduced compared to that from untreated animals (7.73% vs. 17.59% and 6.18% vs. 19.24%respectively) (Fig. 2).

**Figure 2:** TALs of EAC/Dox bearing mice showed Th1 specific response after in vivo administration of CuNG. Flow cytometry. EAC/Dox bearing mice (n = 12) were treated with CuNG (5 mg/kg of body weight), i.m., 7 days following inoculation and 15 days after CuNG administration TALs were isolated from the ascitic fluid of treated and untreated animals as nonadherent population (method described in material and method section). From isolated TALs, CD4 vs. intracellular IFN-γ, IL-4 and TGF-β production were analyzed by flow cytometry and significantly higher percentage of CD4 population of treated group showed positive for IFN-γ (marker for Th1 response). A representative result is presented here for comparison.

### Soluble factors from functionally altered TAMs can skew unresponsive CD4^+^ T cells of untreated EAC/Dox mice towards Th1 type

The conventional role of macrophage in tumor rejection through recognition of tumor antigen and participation in induction of anti-tumor T cell response is changed at the tumor site where it seems to produce elevated levels of immunosuppressive cytokines like IL-10 and TGF-β that effectively attenuate the induction of anti tumor response. We have shown here that single administration of CuNG in EAC/Dox bearing mice was able to alter the functional polarization of TAMs from immunosuppressive to proimmunogenic in nature leading to induction of Th1 type of response at the tumor site. These observations prompted us to investigate whether the soluble mediators derived from CuNG treated TAMs are sufficient to redirect the tumor associated unresponsive CD4^+^ T cells towards Th1 type in the absence of contact dependent signal. To assess this possibility TAMs were isolated from untreated EAC/Dox bearing mice and cultured for 48 h in presence or absence of CuNG. On the other hand TAMs from in vivo CuNG treated mice were cultured in absence of CuNG for 48 h. Following completion of incubation, cell free supernatants were obtained, diluted 2 folds with fresh medium and used to culture CD4^+^ cell enriched TALs. Following 96 h of incubation, cells were harvested and the levels of different Th1 and Th2 cytokine specific mRNA expressions were studied by semi-quantitative RT-PCR using specific primers. We observed that CD4^+^ T cell populations cultured with cell free supernatant of either in vitro CuNG treated TAMs or TAMs from in vivo CuNG treated animals manifested significantly elevated levels of expression of Th1 specific cytokine mRNA (IFN-γ) whereas Th2 specific (IL-4) and suppressive (TGF-β) cytokine mRNA expression levels were undetectable or poorly detectable in these two groups. On the contrary, IL-4 and TGF-β mRNA expressions were found to be significantly higher in the untreated control group (Fig. 3A & B). Similar results were obtained when Th1 and Th2 specific cytokine production by CD4^+^ T cells were analyzed by flow cytometry. CD4^+^ T cell population cultured with cell free supernatant derived from cultures of either in vitro CuNG treated TAMs or TAMs from in vivo CuNG treated mice, induced augmented IFN-γ production from CD4^+^ TALs obtained from untreated EAC/Dox bearing mice. Flow cytometric data (Fig. 3C) also revealed that culture supernatant obtained from in vitro or in vivo CuNG treated TAMs highly reduced the percentage of TGF-β and IL-4 producing CD4^+^ T cells. So both mRNA expression level and intracellular cytokine assay clearly indicate that the pattern of functional cytokine production by a lineage committed CD4^+^ T cells can be modulated in response to its local cytokine microenvironment created by the antigen presenting cells (like TAMs).

**Figure 3:** Culture supernatant of TAMs, treated with CuNG, caused altered cytokines production by TALs. A) RT-PCR. B) Densitometric analysis. C) Flow cytometry. CD4+ T cells were purified from TALs obtained from untreated EAC/Dox bearing mice and cultured for 96 h with cell free supernatant of TAMs obtained from untreated EAC/Dox bearing mice that were either kept untreated for 48 h or treated with CuNG (48 h treatement) in vitro or with cell free supernatant of TAMs (cultured for 48 h in absence of CuNG) obtained from in vivo CuNG (15 days after treatment, i.e., when tumors start regressing prominently) treated EAC/Dox bearing mice. Cytokine profile was analyzed by semi-quantitative RT-PCR. Purified CD4^+^ population from TALs (derived from untreated EAC/Dox bearing mice) cultured without any treatment were used as untreated control. After completion of 96 h of incubation equivalent amount of mRNA (2 µg) from TALs of each experimental group was used for RT-PCR analysis and representative data from three independent experiment is presented (A). In all cases GAPDH was used as housekeeping gene control. Densitometry analysis of mRNA expression of each gene transcript was expressed as a ratio of cytokine mRNA to GAPDH mRNA (B). Intracellular cytokines specific for Th1 (IFN-γ) or Th2 (IL-4) or suppressive (TGF-β) production profile in the above mentioned experimental groups were also analyzed by flow cytometry and representative data of three independent experiments is presented here (C).

### CuNG treated TAMs induce reprogramming of cytokine status of CD4^+^CD25^+^ T cells

CD4^+^CD25^+^FoxP3^+^ (Treg) are well known culprit for creation of immunosuppressive tumor microenvironment via production of high levels of TGF-β [23], [24]. It has previously been shown by us that CuNG treatment in vivo reduces CD4^+^CD25^+^FoxP3^+^ T cells at the tumor site (21). Since under in vitro condition combination of cytokines produced from CuNG treated TAMs can shift the cytokine profile of CD4^+^ TALs from TGF-β producing to IFN-γ producing, therefore we tested whether it can reprogram Treg towards Th1 type. For this purpose sorted CD4^+^CD25^+^ population from TALs of untreated EAC/Dox bearing mice were labeled with CFSE and co-cultured for 96 h with either untreated TAMs or TAMs treated with CuNG in vitro for 48 h. T cells cultured with untreated TAMs maintained their high TGF-β status while cytokine status of T cells cultured with CuNG treated TAMs was reprogrammed to low TGF-β and high IFN-γ (Fig. 4A). Furthermore, majority of the CD25^+^ sorted CD4^+^ cells, when cultured with CuNG treated TAMs, lost their FoxP3 expression vis-à-vis decreasing TGF-β production and increasing IFN-γ generation (Fig. 4B). These cells also lose the characteristic inhibitory property of Treg on proliferation of T cells (Fig. 4C).

**Figure 4:** In vitro CuNG treatment caused reprogramming of Treg. A, B & C) Flow cytometry. CD4^+^CD25^+^ Treg populations were purified from TALs of untreated EAC/Dox bearing mice. (A) Treg cells were labeled with CFSE and then cultured for 96 h with cell free supernatant of TAMs (isolated from untreated EAC/Dox bearing mice) either kept untreated or treated in vitro with CuNG for 48 h. Intracellular IFN-γ and TGF-β production was analyzed with respect to specific isotype control by flow cytometry. Representative data of three independent experiments is shown. (B) Treg cells were cultured for 96 h with supernatant of 48 h culture of untreated or in vitro CuNG treated TAMs and fresh medium (1∶1). Intracellular IFN-γ and TGF-β production versus FoxP3 expression was analyzed with respect to specific isotype control by flow cytometry. Representative data of four independent experiments is shown. (C) Tregs (CD4^+^CD25^+^ cells) isolated from ascitic fluid of untreated EAC/Dox bearing mice were cultured for 96 h in presence of cell-free supernatants from 48 h cultures of untreated or CuNG treated TAMs (culture supernatant: fresh medium being 1∶1). Now, these cells were washed and cultured with CFSE loaded CD4^+^ T cells isolated from inguinal and axillary lymph nodes of normal mice (Treg and CD4^+^ T cells were taken in a proportion of 1∶5) for 96 h. Fluorescence levels of CFSE were measured by flow cytometry. Proliferation of normal CD4^+^ T cells either in the presence or absence of Treg cells were also analyzed by CFSE fluorescence level. Representative data of 3 independent experiments is presented here.

### Redirection of the tumor associated CD4^+^ T cells towards Th1 type can be accounted for by CuNG mediated altered level of IL-10 and IL-12 production from TAMs

It is well evident from Fig. 1B that CuNG treatment caused alteration in the levels of IL-10 and IL-12 production by TAMs but did not completely abrogate the IL-10 production. This observation made us curious to further investigate whether the combination of low level of IL-10 and high level of IL-12 that we obtained with TAMs after CuNG treatment would have the same potential as IL-12 alone to make the decision for the generation of the Th1 response. To test this hypothesis, CD4^+^ TAL from untreated EAC/Dox bearing mice were cultured in the presence of either recombinant IL-10 (rIL-10) or IL-12 (rIL-12) alone or with a combination of rIL-10 and rIL-12 for at least 96 h. The doses of rIL-10 and rIL-12 applied corresponded to those obtained from the ELISA data of IL-10 and IL-12 production by either untreated or in vitro CuNG treated TAMs. Both mRNA expression study (Fig. 5A & B) and intracellular cytokines production assay (Fig. 5C) indicated that CD4^+^ T cells population cultured in the presence of 0.35 ng/ml of rIL-10 and 2.7 ng/ml of rIL-12 showed a significant up-regulation in production of IFN-γ similar to CD4^+^ TALs treated with only a single high dose of rIL-12. On the other hand, CD4^+^ TALs stimulated in the presence of 1.3 ng/ml of rIL-10 and 0.2 ng/ml of rIL-12 (amount similar to the IL-10 and IL-12 obtained from untreated TAMs), did not show any remarkable change in cytokine production pattern from that we observed in case of single high dose of rIL-10 treated or untreated control group.

**Figure 5:** Combination of high IL-12 and low IL-10 can skew induction of Th1 response. A) RT-PCR. B) Densitometric analysis. C, D, E & F) Flow cytometry. CD4^+^ population from TALs (obtained from untreated EAC/Dox bearing mice) was purified and challenged either with single or combine dose of recombinant IL-12 and IL-10 and cultured for 96 h. Purified CD4^+^ population from TALs derived from untreated EAC/Dox bearing mice, cultured without any treatment was taken as untreated control. Equivalent amount of mRNA (2 µg) from each experimental group was used for semi-quantitative RT-PCR analysis and in all cases GAPDH was used as housekeeping gene control (A). Densitometry analysis of mRNA expression of each gene transcript was expressed as a ratio of cytokine mRNA to GAPDH mRNA (B). Intracellular cytokines specific for Th1 (IFN-γ) or Th2 (IL-4) or suppressive (TGF-β) production profile in the above mentioned experimental groups were also analyzed by flow cytometry and a representative data is shown (C). CD4+ TALs were co-cultured with untreated TAMs or CuNG treated TAMs either unfixed or fixed with paraformaldehyde or CuNG treated fixed TAMs along with high rIL-12 and low rIL-10. In some cases CD4+ TALs and CuNG treated unfixed TAMs were separated by transwell insert (0.45 µ Meter pore) in culture. After 96 h of culture intracellular IFN-γ and TGF-β production pattern were studied by flow cytometry (D). Mean fluorescence intensity for IFN-γ (Fig. 5E) and TGF-β (Fig. 5F) production by these experimental groups were also analyzed from the flow cytometric statistical data and represented graphically. Representative data from three independent experiments is presented.

Interestingly it is also evident from dot plot analysis of flow cytometry data (Fig. 5C) that the percentage of IFN-γ positive cells among CD4^+^ TALs was higher when cultured in the presence of combination of high rIL-12 and low rIL-10 compared to the high rIL-12 alone (54.42% vs. 36.89%). Interestingly, CuNG treated TAMs, when fixed with paraformaldehyde could not increase IFN-γ production or decrease TGF-β generation in CD4^+^ TALs. However, when a combination of low rIL-10 and high rIL-12 was introduced in this system, TALs were reprogrammed (Fig. 5D). Moreover, co-culture of CuNG treated TAMs and CD4^+^ TALs did not significantly increase the level of reprogramming (Fig. 5D). These results indicate that reprogramming of TALs strongly depends on soluble agents (high IL-12 and low IL-10) released from reprogrammed TAMs. However, the cause of lower percentage of IFN-γ producing TALs following rIL-12 treatment alone compared to that following treatment with high rIL-12 and low rIL-10 remained unanswered. To explain this differential response we reasoned that the combination of high rIL-12 and low rIL-10 might block the death of T cells.

### Presence of small amount of IL-10 in association with IL-12 delayed the death of Th1 population

Several reports are corroborating the fact that high level of IFN-γ produced by the Th1 population mediates its own apoptosis by up-regulating both Fas and Fas-L expression [25], [26], [27], [28]. Recently a differential role of IL-10 as an anti-apoptotic mediator protecting the mouse intestinal epithelial cells from IFN-γ or TNF-α mediated apoptosis by diminishing the Fas expression has been shown [29]. These findings prompted us to investigate whether the presence of low level of rIL-10 in combination with high rIL-12 could prolong the Th1 response by interfering with its self-killing mechanism. To address the issue of involvement of IL-10 in prolonging Th1 response, we cultured CD4^+^ T cells obtained from TALs of untreated EAC/Dox bearing mice either with a single high dose or different combination of rIL-10 and/or rIL-12 for 5 days. Cell death was quantified by means of PI/Annexin V-FITC. It was observed that rIL-12 alone induced high levels of apoptosis while a combination of low rIL-10 and high rIL-12 protected CD4^+^ T cells from undergoing apoptosis (Fig. 6A). This apoptotic process was found to be associated with caspase 3 activation. An active caspase 3 level in each experimental group was represented by the fluorescence intensity of the cleaved fluoregenic AMC liberated due to cleavage of Ac-DEVD-AMC by active caspase 3. Caspase 3 assay clearly indicates (Fig. 6B) that intensity of active caspase 3 levels in the high rIL-12 treated group increased much faster than high rIL-12 plus low rIL-10 treated group (15.663±0.57 vs. 15.107±1.06 at 72 h, 21.755±0.74 vs. 16.090±0.61 at 96 h and 27.223±0.60 vs. 18.414±0.36 at 120 h respectively). Addition of cell free supernatant derived from 48 h culture of both in vitro CuNG treated TAMs (originally isolated from untreated animals) and in vivo CuNG treated TAMs (obtained from in vivo CuNG treated animals) in the culture of CD4^+^ TALs from untreated animals resulted in restricted increase of caspase 3 activity (14.16±0.89 at 72 h, 17.59±0.46 at 96 h and 20.36±0.86 at 120 h and 15.65±0.46 at 72 h, 16.64±0.28 at 96 h and 18.93±0.53 at 120 h respectively) while neutralization of IL-10 in corresponding sets resulted in rapid increase of caspase 3 activity (16.33±0.76 at 72 h, 23.22±0.94 at 96 h and 29.65±0.71 at 120 h and 15.23±0.49 at 72 h, 20.99±0.49 at 96 h and 28.02±0.49 at 120 h respectively) (Fig. 6B).

**Figure 6:** Presence of small amount of IL-10 prolonged Th1 response by delaying T cells apoptosis. A) Flow cytometry. B) Fluorometric analysis. C & D) Flow cytometry. Purified CD4^+^ population from TALs of untreated EAC/Dox bearing mice cultured in the presence of either only rIL-12 or the combination of high rIL-12 (2.7 ng/ml) and low rIL-10 (0.35 ng/ml) or the culture supernatant of in vitro CuNG treated (48 h of CuNG treatment) TAMs or IL-10 neutralized culture supernatant of in vitro CuNG treated (48 h of CuNG treatment) TAMs or 48 h of culture supernatant from in vivo CuNG treated TAMs or IL-10 neutralized culture supernatant of in vivo CuNG treated TAMs, for 72 h, 96 h and 120 h. Purified CD4^+^ population without any treatment was taken as untreated control. Levels of apoptosis were estimated by PI/Annexin V-FITC staining and flow cytometry. Representative data of 3 independent experiments is presented here (A). Purified CD4^+^ population pre-treated with H2O2 for 30 mins was taken as positive control for active caspase 3 level (Mean fluorescence intensity value of H2O2 control was 39.25±0.67 that was taken as 100% for active caspase 3 level). In each experimental group active caspase 3 levels was represented by % of H_2_O_2_ positive control. Results presented are of 4 independent experiments (B). Expression of Fas by CD4^+^ population of above mentioned experimental groups were also analyzed by flow cytometry. Cells were labeled with Abs specific for CD4 and for surface Fas or with specific isotype Abs and immunofluorescence analysis was performed. Representative result of 4 independent experiments is presented (C). CD4^+^ TALs were cultured with or without different combinations of rIL-12 and rIL-10 in absence or presence of neutralizing antibody against IFN-γ for 72 h. Fas expression was studied by flow cytometry and representative data of 3 independent experiments is presented here (D).

Next, to decipher the mechanism underlying IL-10 mediated inhibition of Th1 polarized CD4^+^ T cell death we studied the Fas expression in the above population. To assess this possibility levels of Fas expression by CD4^+^ T cells of untreated EAC/Dox bearing mice cultured either with combination of high rIL-12 and low rIL-10 or high rIL-12 alone, were analyzed at 72 h, 96 h and 120 h. It was evident from the Fig. 6C that initially at 72 h CD4^+^ T cells cultured in the presence of high dose of rIL-12 alone showed Fas positive population comparable to that of CD4^+^ T cells cultured with a combination of high rIL-12 and low rIL-10. However, at 96 h and 120 h positive population for Fas expression was significantly higher in CD4^+^ T cells cultured in the presence of high dose of rIL-12 alone. Addition of cell free supernatant either from 48 h culture of in vitro CuNG treated TAMs or 48 h culture of TAMs from in vivo CuNG treated animals, at a ratio of 1∶1 with fresh medium in culture of TALs obtained from untreated animals resulted in low levels of Fas expression while neutralization of IL-10 in corresponding sets resulted in increased Fas expression (Fig. 6C). These data clearly indicate that presence of low level of rIL-10 in association with high rIL-12 do not interfere with the normal function of IL-12 in inducing Th1 response although delayed apoptosis by diminishing Fas expression thus prolonged the Th1 response. The ratio of rIL-10 and rIL-12 in this combination was almost 1∶8, as obtained by ELISA. So we tested other combinations like 1∶4, 1∶12, 1∶16 and rIL-12 only along with this combination. It was observed that 1∶4 and 1∶8 were the best combinations in terms of low Fas expression (Fig. 6D, upper panel) while with 1∶8, IFN-γ expression was much higher than 1∶4 (data not shown). Neutralization of IFN-γ yielded low levels of Fas expression in all cases (Fig. 6D, lower panel) indicating that IL-12 mediated IFN-γ generation caused Fas expression and T cell death. Thus, IL-12 is the key factor for reprogramming CD4^+^ cells towards IFN-γ producing Th1 type as well as inducing T cell death through IFN-γ production.

### CuNG treatment in vitro reduces the immunosuppressive cytokines and induces IL-12 generation in blood monocytes of patients with metastatic cancers

Next we have tried to extrapolate our experimental data under clinical condition to see whether CuNG can modulate peripheral blood monocytes from patients to produce similar effect. PBMC isolated from patients with drug-resistant metastatic cancers was treated in vitro with CuNG. After 72 h, CD14^+^ adherent population was tested for the cytokine status. Untreated CD14^+^ cells exhibited an alternative activation status marked by high levels of TGF-β and IL10. Interestingly, following CuNG treatment, CD14^+^ cells exhibited very low levels of TGF-β, lowered IL-10 and high levels of IL-12 (Fig. 7).

**Figure 7:** Treatment of CuNG upregulates IL-12 production by adherent population of PBMC from different cancer patients sample. Flow cytometry. PBMC from different cancer patients were isolated and only adherent population was either treated with CuNG (2.5 µg/ml) or kept untreated for 48 hr. Cells was labeled with Abs specific for surface CD14 and intracellular IL-10 or IL-12 or TGF-β and analyzed by flow cytometry.

## Discussion

Present study establishes a new paradigm whereby the modulation in regulatory cytokine production pattern of tumor associated macrophages (TAMs) by the copper chelate CuNG is an effective strategy to remodel the local cytokines milieu in the tumor microenvironment. This plays a pivotal role in skewing unresponsive and suppressive CD4^+^ T cell populations towards Th1 type in EAC/Dox bearing mice.

Macrophages are the most versatile cells population and are capable of changing their functional polarization in response to the growth factors or cytokines being released in their microenvironment [30], [31]. Cytokine milieu profoundly affects the functional polarization of the macrophages [31], [32]. Several studies indicate that tumor derived factors educate the newly recruited monocytes towards TAMs, which become immunosuppressive in nature [6], [7]. There is a symbiotic relationship between TAMs and cancer cells, where cancer cells attract TAMs and sustain their survival and TAMs in turn produce various growth and proangiogenic factors that promote tumor progression and metastasis [8], [33], [34] as well as effectively thwart the induction of protective anti-tumor response [6]. However, evidences suggest that TAMs retain functional plasticity and could be converted to nonsuppressive and anti-tumorogenic type by creating appropriate cytokine microenvironment [12]. Stout et al. showed that in the presence of IL-12 TAMs rapidly alter their functional phenotype from tumor-supportive and immunosuppressive to inflammatory [12]. In our study we have showed that a novel copper chelate, CuNG, possesses the potential to alter the immunosuppressive phenotype of TAMs by reprogramming its proinflammatory (IL-12) versus immumosuppressive (IL-10 and TGF-β) cytokine production pattern. Current study also demonstrated that both in vitro and in vivo application of CuNG evoked a robust IL-12 and diminished IL-10 and TGF-β production by TAMs and thereby polarize its functional phenotype towards inflammatory.

The induction of Th1 response highly depends on the critical level of the two regulatory cytokines, IL-10 and IL-12 [35], [36]. IL-10 inhibits important aspects of cell-mediated immunity whereas IL-12 induces type 1 cytokine production and effective anti-tumor cell mediated response [37], [38]. IL-10 overproduction by TAMs at the tumor site has been implicated in tumor mediated immune suppression [39]. It has also been found that transgenic mice over expressing IL-10 under the control of IL-2 promoter were unable to restrict the progression of immunogenic tumor whereas applying anti IL-10 mAbs in these mice restored the in vivo antitumor response [40]. In addition to IL-10, high TGF-β secretion by TAMs at the tumor microenvironment seems to play a potent immunosuppressive role by inhibiting T cell activation, proliferation and differentiation [11], [33], [39]. In contrast, IL-12, which stimulates Th1-dominant immunity in vivo, was shown to have strong in vivo anti-tumor activity [14], [38]. In our study we have shown that CuNG caused reduced IL-10 and TGF-β and augmented IL-12 production by TAMs at the tumor site. Elevated levels of IL-12 production by TAMs after CuNG treatment altered the cytokine balance at the tumor site and established a beneficial cytokine microenvironment that efficiently countered the immunosuppressive influence as well as skewed the unresponsive CD4^+^ T cells population towards Th1 type. Moreover, this reprogramming effect was found to be quite independent of cell-cell contact.

Persistence of Th1 response is greatly inhibited due to self-killing of T cells due to over production of IFN-γ. This remains a major obstacle for successful tumor immunotherapy. Addition of IL-12 results in hugely elevated levels of IFN-γ [41], which limits T cell survival [42] and shortens Th1 response. Addition of IFN-γ induces a short-lived tumorocidal effect followed by immunosuppression and aggressive tumor growth, limiting its use as an immunotherapeutic agent [42]. High expression of death receptors and caspase 3 in Th1 cells make them prone to apoptosis [25]–[28]. Our study demonstrates that both in vivo and in vitro CuNG treated TAMs maintained a stable balance between IL-10 and IL-12 production where IL-12 levels were ∼8 folds higher than IL-10. This critical balance between these two cytokines was sufficient enough to induce Th1 response, as well as, the presence of small amount of IL-10 limits the self killing mechanism of Th1 cells and thereby prolonged its persistence. Moreover, CuNG treated TAMs could modulate TGFβ producing CD4^+^CD25^+^ T cells toward IFNγ producing T cells with concomitant decrease in the level of FoxP3 expression, indicating that Treg can be reprogrammed toward Th1 phenotype. Similar modulation of peripheral blood monocytes from chemo and/or radiotherapy refractory cancer patients from immunosuppressive to pro-inflammatory status could be achieved by in vitro CuNG treatment. This could also modulate Th2 type response to Th1 response (data not shown).

The mechanisms underlying modulation of cytokine behavior of TAM by this copper complex is yet to be deciphered and the role of modulation of redox status cannot be ruled out [43]. The current study suggests that CuNG treatment induced a sustained generation of ROS. Inhibition of this ROS with anti-oxidant reversed the cytokine generation status of CuNG-treated TAMs toward untreated TAMs. Ongoing studies in this direction point towards the complex interplay between intracellular signaling events and the increase in reduced glutathione (GSH) level in late hour of CuNG treatment following its initial depletion (2 h) in the context of pattern of modulation of cytokine profile in macrophages (our unpublished observation).

In summary, we critically evaluated the anti tumor efficacy of the novel copper chelate (CuNG) for its potential role of modulating TAMs and thereby inducing protective anti tumorogenic Th1 response. Earlier study with CuNG explored its immunomodulatory effects especially against drug resistant tumors [21]. Here we demonstrated that CuNG causes immune modulation in drug resistant cancer bearing individuals by altering functional cytokine pattern of TAMs to establish a proper immune surveillance at the tumor site. These data indicate that CuNG may be used clinically for immunotherapy of different types of drug resistance cancers.

## Materials and Methods

### Reagents

Penicillin, Streptomycin was purchased from Sigma (USA). Recombinant murine IL-10, IL-12, opt EIA kit for assay of murine cytokines, anti-mouse IFN-γ, IL-10, IL-4, FITC conjugated IL-12 mAb, anti-mouse TGF-β, PE conjugated TNF-α mAb and all human reactive antibodies were purchased from BD Bioscience/BD Pharmingen (USA). Anti CD5 and CD19, F4/80 biotin conjugated mAb (murine) were obtained from eBioscience (USA). The cell culture medium RPMI-1640 and FCS were purchased from Gibco, Invitrogen (USA).

### Animals and Cell lines

Swiss albino mice, obtained from National Institute of Nutrition (Hyderabad, India) and maintained in the institute animal facilities, were used for experimental purpose with prior approval of the Institutional Animal Ethics committee. EAC/Dox, which is resistant against doxorubicin, cisplatin, cyclophosphamide and vinblastine were developed and maintained according to the previously described methods. [44].

### Treatment of Animals

EAC/Dox bearing mice were kept either untreated or treated with a single dose of CuNG (5 mg/kg of body weight) 7 days following peritoneal inoculation with 1×10^6^ EAC/Dox cells obtained from EAC/Dox bearing mice treated with Dox (48 hrs before acquisition of cells) [21].

### Cell isolation and purification

#### Isolation of Tumor associated macrophages (TAM)

Total ascitic fluid was drawn and kept at standing position in a 50 ml sterile tube for at least 2 hrs for settling down the tumor cells and then clear fluid from the upper zone was collected. TAMs were isolated from that clear fluid first by negative selection with anti CD5 and anti CD19 and then by positive selection with anti F4/80 using BD IMagnet system (BD Bioscience) according to the manufacturer's protocol and resuspended in RPMI-1640 containing 10% FCS. Flow cytometric data revealed that purity of the separated population was >90%.

#### Isolation of tumor associated lymphocytes (TAL) and purification of CD4^+^ T cells from TAL

For isolation of TALs, total ascitic fluid was drawn, the upper clear zone of the ascitic fluid that remained after the tumor cells settled down was collected and centrifuged and the pellet was resuspended in RPMI-1640 containing 10% FBS and plated over the 90 mm plastic tissue culture plates and kept for at least ∼4 hrs at 37°C under 5% CO_2_ in air to allow the attachment of adherent cells. Nonadherent cells ( TALs, 95% lymphocytes) were subsequently removed by aspiration, harvested by centrifugation and resuspended in RPMI-1640 containing 10% FCS. In some cases CD4^+^ populations from TALs were purified by single positive selection with anti CD4-DM particle (BD Biosciences) or Treg were isolated from TAL using Treg isolation kit (BD Biosciences) using BD IMagnet system according to the manufacturer's protocol.

### Treatment of TAMs and assay of different cytokines production by flow cytometry and ELISA and estimation of ROS generation

TAMs from either treated or untreated group were incubated with anti-F4/80-FITC or PE conjugated monoclonal antibody for 45 min at 4°C. After extensive washing, cells were then fixed, and permeabilized and stained with anti IL-12- FITC, anti IL-10- PE and anti TGF-β- FITC mAbs or corresponding isotype controls as described previously [21] and analyzed by flow cytometer (FACS calibur, BD).

TAMs from untreated EAC/Dox bearing mice were plated (2×10^6^ cells/ml) in 24 wells plate in the presence or absence of CuNG (2.5 µg/ml). Supernatants were collected after 12 h, 24 h and 48 h and assayed in triplicate for the production of IL-10, IL-12 and TGF-β using opt EIA kit (ELISA kit from BD Bioscience) according to the manufacturer's protocol.

Reactive oxygen species (ROS) generation by differentially treated TAMs was measured using dichlorofluorescein diacetate (DCF-DA) using standard protocol described previously [45], [46].

### Treatment of CD4^+^ T cells and Treg of untreated EAC/Dox bearing mice in vitro

The purified total CD4^+^ population from TALs of untreated mice were plated (2×10^6^ cell/ml) and cultured with or with out CuNG (2.5 µg/ml) for 24 h, 48 h and 72 h and the supernatant was taken and assayed in triplicate for the production of IFN-γ using optEIA kit (ELISA kit from BD Bioscience) according to the manufacturer's protocol. In some cases the purified total CD4^+^ TAL were plated (2×10^6^ cell/500 µl) in presence of 500 µl of culture supernatant obtained after culturing TAMs derived either from in vivo CuNG treated mice or untreated EAC/Dox bearing mice treated in vitro with CuNG (48 h of treatment). In every case TAMs concentration was 2×10^5^ cell/ml. In some cases different doses of recombinant IL-10 and IL-12 either individually of in combination was applied on CD4^+^ T cells (2×10^6^ cell/ml). In some experiments CD4^+^CD25^+^ cells (Treg; 1×10^6^ cell/ml) isolated from tumor site of untreated EAC/Dox mice (≥80% FoxP3^+^) were first labeled with CFSE (5 µM/ml) and then cultured in AIM V medium either with culture supernatant of in vitro CuNG (48 h of CuNG treatment) treated TAMs or untreated TAMs. For stimulation of CD4^+^ T cells anti-CD3 antibody (5 µg/ml) and anti CD-28 (1 µg/ml) antibody was also applied in this culture medium and incubated at 37°C with 5%CO_2_ 95%air atmosphere condition. After 96 h of incubation non-adherent populations (90–95% lymphocytes) were collected by centrifugation at 500 g for 10 mins for performing further experiments. For neutralization of IL-10, 100 µg/mL neutralizing anti-IL-10 antibody was used.

### Assay of different cytokines production from CD4^+^ T cells by semi-quantitative RT-PCR and flow cytometry

For assay of different cytokines by semi quantitative RT-PCR RNA was extracted from purified CD4^+^ T cells using NucleoSpin RNA II kit (Machery-Nagel) and reverse transcribed using RETROscript (Ambion). Primers specific for murine TGF-β (sense, CTTTAGGAAGGACCTGGGTT; antisense CAGGAGCGCACAAT-CATGTT), TNF-α (sense ATGAGCACAGAAAGCATGATC; antisense TACAGGCTTGTCACTCGA ATT), IFN-γ (sense CTCAAGTGGCATAGATGTGGA; antisense GACCTCAAACTTGGCAATACTC), IL-4 (sense GTCATCCTGCTCTTCTTTCTC; antisense ATGCTCTTTAGGCTTTCCAG), IL-10 (sense ACTACCAAAGCCACAAAGCAG; antisense AAGGAGTCGGTTAGCAGTATG) and GAPDH (sense CCCACAGTAAATTCAACGGCAC; antisense CATTGGGGTTAGGAACACGGA) were used with 2 µg of sample cDNA and amplified with Taq polymerase (Promega) using a Thermal Cycler (Applied Biosystem). For intracellular cytokines staining of CD4^+^ population the above mentioned staining protocol were used. In brief CD4^+^ population from different experimental groups were labeled with anti CD4 FITC or PE and intracellular anti IFN-γ FITC or anti IL-4 PE or anti TGF-β PE and immunoflorescence analysis was performed by using FACScaliber (BD Biosciences) with CellQuest software.

### Caspase assay and Fas expression study of Th1 polarized CD^+^ T cells

Purified CD4^+^ T cells from TALs of untreated EAC/Dox bearing mice were cultured either with a single high dose of rIL-12 (2.7 ng/ml) or combination of high rIL-12 (2.7 ng/ml) and low rIL-10 (0.35 ng/ml) or culture supernatant of in vitro CuNG (48 h of CuNG treatment) treated TAMs or IL-10 neutralized culture supernatant of in vitro CuNG (48 h of CuNG treatment) treated TAMs or IL-10 neutralized culture supernatant of in vivo CuNG (15 days of CuNG treatment) treated TAMs for 72 h, 96 h and 120 h. Purified CD4^+^ population without any treatment was taken as untreated control. 30 mins pretreatment with H_2_O_2_ (500 µM/ml) was considered as positive control. An active caspase 3 level was assayed by using caspase 3 assay kit (BD Pharmingen) according to the manufacturer's protocol using spectrofluorimeter (Varian). In these groups CD4^+^ population vs. Fas expression was also studied by flow cytometry.

### Cytokine assay of adherent population of PBMC isolated from different cancer patients

Leftover excess of blood drawn for routine examination of cancer patients refractory to various chemotherapeutics (certified by the Department of Surgical Oncology and Medical Oncology, Hospital Unit, Chittaranjan National Cancer Institute) were collected as sample from the Department of Clinical Biochemistry, Hospital Unit, Chittaranjan National Cancer Institute. Patient profile is given in Table 1. PBMC were isolated by Histopaque™ (Sigma). Adherent population from PBMC was isolated and either kept untreated of treated with CuNG (2.5 µg/ml) for 48 h. Intracellular cytokines were assayed by above mentioned protocol, in brief, adherent cells were scraped off from the plate and labeled with anti human CD14 FITC and intracellular anti human IL-10 PE or anti human IL-12 PE or anti human TGF-β PE and analysis was performed using FACScaliber (BD Biosciences) with CellQuest software.

**Table 1:** Patient profiles.

Patient	Age (years)	Sex	Tumor type	Remarks
1	66	F	CA breast	Brain metastasis; unresponsive to radiotherapy, 5-FU and anthracyclin (Epirubicin).
2	50	M	CA lung	Adrenal metastasis; unresponsive to Pacitaxel, cisplatin and radiotherapy.
3	35	F	CA rectum	Liver metastasis; unresponsive to 5-FU and radiotherapy.
4	45	M	CA cheek	Unresponsive to cisplatin, bleomycin and MTX.

### Statistical analysis

Each experiment was done three to five times and results were expressed as mean±SE and Student's t test for significance was done and P<0.01 was considered significant. Flow cytometric data show representative data of at least three independent experiments.
